RETRACTED

# Clinical Efficacy and Safety Analysis of PD-1/PD-L1 Inhibitor vs. Chemotherapy in the Treatment of Advanced Non-Small-Cell Lung Cancer: A Systematic Review and Meta-Analysis

**DOI:** 10.1155/2022/9500319

**Published:** 2022-06-25

**Authors:** Wei-wei Guo, Tian-wei Zhang, Bin-liang Wang, Li-qun Mao, Xiao-bo Li

**Affiliations:** Department of Respiratory and Critical Care Medicine, Taizhou First People's Hospital, Taizhou City, Zhejiang Province, China 318020

## Abstract

**Objective:**

To systematically evaluate the efficacy and safety of pembrolizumab (PD-1/PD-L inhibitor) and adjuvant chemotherapy to treat NSCLC and provide evidence-based reference for clinical use.

**Methods:**

By searching the Cochrane Library, EMBASE, PubMed, and Web of Science, according to the inclusion criteria, literature selection, data extraction, and quality evaluation were carried out for the included literature. The *I*^2^ test was used to evaluate heterogeneity between studies, and the meta-analysis was performed using RevMan 5.3 software provided by Cochrane.

**Results:**

Finally, 14 relevant documents meeting the standards were included. It is a statistical difference in one-year survival rate [OR = 1.50, 95% CI (1.28, 1.76), *P* < 0.00001, *I*^2^ = 0%, *Z* = 4.99]; overall response rate[OR =1.57, 95% CI (1.29, 1.90), *P* < 0.00001, *I*^2^ = 0%, *Z* = 4.58]; progression-free survival [OR = 2.99, 95% CI (2.29, 3.91), *P* < 0.00001, *I*^2^ = 26%, *Z* = 8.00]; and overall survival [OR = 1.38, 95% CI (1.07, 1.78), *P* = 0.01, *I*^2^ = 46%, *Z* = 2.50] and reduces the incidence of adverse drug reactions [OR = 2.54, 95% CI (1.99, 3.25), *P* < 0.00001, *I*^2^ = 69%, *Z* = 7.43].

**Conclusion:**

Pembrolizumab adjuvant chemotherapy is effective in the treatment of advanced NSCLC, but attention should be paid to the occurrence of adverse reactions in clinical. Due to the limitations of the methodology included in the study, this conclusion required more validation of large-sample RCT.

## 1. Introduction

In recent years, the research achievements of immunotherapy are outstanding, and a number of clinical trials are reported frequently [1]. Lung cancer is one of the most deadly malignancies, with a 5-year survival rate of less than 18%, among which non-small-cell lung cancer (NSCLC) accounts for 85% of the total. The treatment of lung cancer takes a period of 10 years, from the era of chemotherapy, antivascular therapy, and targeted therapy to the current era of immunotherapy [2–4]. With the deepening of the research on the mechanism of tumor immune escape, it is found that negative immune regulation of some immune checkpoints plays an important role in the formation of tumor. Programmed cell death 1 (PD-1) and PD-1 ligand (PD-L1) enhance the resistance of tumor microenvironment to normal immunity through immune escape, inhibition of immune response, avoidance of killing, and elimination [5]. The efficacy and safety of immunosuppressants targeting the PD-1/PD-L1 pathway have been confirmed in large clinical trials of the local late maintenance therapy, late second-line therapy, and late first-line therapy of NSCLC [6]. In 2020, a multicenter, open Phase III trial test also verified the effect [7]. It is only 20% efficient and has an overall survival period of only 8 to 10 months [8]. EGFR(+) is found in about 80% of NSCLC patients, so the targeted treatment regimens acting on EGFR have become a new direction for NSCLC therapy [9]. Pembrolizumab suppresses epidermal growth factor activation and the conduction of downstream intracellular signaling. In 2009, pembrolizumab was added to the first-line treatment with the NCCN guidelines for relapse and metastatic NSCLC regimen. However, pembrolizumab has not been approved for any first-line and maintenance therapy for NSCLC in China. The US FDA approved only pembrolizumab for the treatment of metastatic colorectal and head and neck cancers and did not for the treatment of NSCLC. NSCLC has a short survival period and a high mortality rate, and it is difficult for the traditional chemotherapy regimen to achieve a better therapeutic effect. Targeted treatment has gradually become a major trend to treat NSCLC [10]. At present, pembrolizumab has entered phase clinical trials for NSCLC, but pembrolizumab has not been granted for any first-line and maintenance treatment of NSCLC, and pembrolizumab is not sure to benefit NSCLC patients.

RETRACTED

Therefore, in this study, the clinical efficacy and safety of pembrolizumab adjuvant chemotherapy were compared according to the Cochrane systematic evaluation method, providing a scientific basis for first-line use of pembrolizumab for advanced NSCLC.

## 2. Materials and Methods

### 2.1. Search Strategy

Using the literature tracing approach, we carefully searched PubMed and EMBASE and gathered relevant literatures published both at home and abroad. The following are the keywords used: pembrolizumab, lung cancer, chemotherapy, PD-1/PD-L1, and others. The retrieval date ranges from the moment the database was created to December 31, 2021. At the same time, included references were tracked, and relevant conference papers were manually retrieved to recover unretrieved material, and the literature gathered was separately appraised by the two reviewers (Figure 1).

### 2.2. Research Type

RCTS have been published at both home and abroad, whether blind or not.

RETRACTED

### 2.3. Research Objects

The following are the research objects: (1) age 18 with no gender restriction; (2) pathological diagnosis of NSCLC; (3) stage II/IV NSCLC confirmed by imaging or other clinical examinations; (4) Karnofsky score of 60 or ECOG score of 0-2; and (5) no absolute contraindication to chemotherapy prior to treatment and no obvious abnormality of liver and kidney function, hematology, or electrocardiogram

### 2.4. Intervention Methods

The experimental group was given pembrolizumab+platinum-based chemotherapy, while the control group was given only platinum-based chemotherapy. Dose and course of pembrolizumab and other chemotherapy drugs are not limited.

### 2.5. Outcome Indicators

Therapeutic indexes include 1-year survival rate (1 year after randomization cases/total number of cases of survival); complete remission rate (complete response cases/total number of cases, complete response referring to the lumps disappearing completely, and duration of 1 month or more); partial remission rate (relieving some cases/total number of cases, partial response refers to the mass decrease 50% or higher, and duration ≥ 1 month); and total response rate [ORR (total response+partial response)/total response]. Safety indicators included the incidence of anemia, thrombocytopenia, leukopenia, rash, dyspnea, infusion response, vomiting, fever, and mortality.

### 2.6. Exclusion Criteria

The following are the exclusion criteria: (1) patients with a history of small-cell lung cancer or other malignant tumors; (2) patients with severe impairment of heart, liver, or kidney function; (3) a prior history of chemotherapy; and (4) a prior history of EGFR-targeted drugs or monoclonal antibodies with poorly controlled BMS.

### 2.7. Literature Quality Assessment

Two researchers independently extracted data and cross-checked to ensure the accuracy of the data. The quality evaluation method of RCT was based on the standard of Cochrane Handbook 5.0.2 (Figures 2 and 3).

### 2.8. Statistical Analysis

RevMan 5.2 statistical software was used for meta-analysis, while for continuous variables, Weighted Mean Difference (WMD) and 95% confidence interval (CI) were used to represent the effect size. A *χ*^2^ test was used for hypothesis testing to determine the heterogeneity among the results of each included study, and *P* < 0.05 was considered statistically significantly different. The studies without statistical heterogeneity (*P* > 0.1, *I*^2^ < 50%) were analyzed by a fixed-effects model. For studies with statistical heterogeneity (*P* < 0.1, *I*^2^ ≥ 50%), a random-effects model was used for pooled analysis.

## 3. Result

### 3.1. Literature Retrieval Results and Included Research Characteristics

A total of 369 literatures were obtained in the preliminary examination, and 259 duplicated literatures were excluded. 96 literatures were screened out after reading the title and abstract, and 14 literatures were included after reading the full text. Figure 1 is the literature retrieval and screening process (Table 1).

RETRACTED

### 3.2. One-Year Survival Rate

The HR value of one-year survival rate and 95% confidence interval were combined, and there was no statistical heterogeneity among the included studies (*I*^2^ = 0%, *P* < 0.00001), and a fixed-effects model was used for meta-analysis. Therefore, there was a statistical difference in one-year survival rate between two groups [OR = 1.50, 95%CI (1.28, 1.76), *P* < 0.00001, *I*^2^ = 0%, *Z* = 4.99] (Figure 4).

### 3.3. Overall Response Rate(ORR)

The HR value of overall response rate and 95% confidence interval were combined, and there was no statistical heterogeneity among the included studies (*I*^2^ = 0%, *P* < 0.00001), and a fixed-effects model was used for meta-analysis. Therefore, there was a statistical difference in overall response rate between two groups [OR = 1.57, 95%CI (1.29, 1.90), *P* < 0.00001, *I*^2^ = 0%, *Z* = 4.58] (Figure 5).

### 3.4. Progression-Free Survival

The HR value of progression-free survival and 95% confidence interval were combined, and there was no statistical heterogeneity among the included studies (*I*^2^ = 26%, *P* < 0.00001), and a fixed-effects model was used for meta-analysis. Therefore, there was a statistical difference in progression-free survival between two groups [OR = 2.99, 95%CI (2.29, 3.91), *P* < 0.00001, *I*^2^ = 26%, *Z* = 8.00] (Figure 6).

### 3.5. Overall Survival (OS)

The HR value of overall survival and 95% confidence interval were combined, and there was no statistical heterogeneity among the included studies (*I*^2^ = 46%, *P* = 0.01), and a fixed-effects model was used for meta-analysis. Therefore, there was a statistical difference in overall survival between two groups [OR = 1.38, 95%CI (1.07, 1.78), *P* = 0.01, *I*^2^ = 46%, *Z* = 2.50] (Figure 7).

### 3.6. Incidence of Coincidences

The HR value of incidence of coincidences and 95% confidence interval were combined, and there was no statistical heterogeneity among the included studies (*I*^2^ = 69%, *P* < 0.00001), and a fixed-effects model was used for meta-analysis. Therefore, there was a statistical difference in incidence of coincidences between two groups [OR = 2.54, 95%CI (1.99, 3.25), *P* < 0.00001, *I*^2^ = 69%, *Z* = 7.43] (Figure 8).

## 4. Discussion

At present, lung cancer remains the main cause of cancer-related death worldwide, ranking first in cancer mortality in men and second in women [25, 26]. According to the WHO statistics, there were about 2.1 million new lung cancer cases and 1.8 million cancer deaths in 2018, accounting for 11.6% of the total new cancer cases and 18.4% of the total cancer deaths, respectively, and the 5-year survival rate was only 10% to 20% [27]. In recent years, immunotherapy has become an emerging hot spot in lung cancer treatment, in which programmed cell death receptor1 (PD-1) and immunocheckpoint inhibitors represented by PD-L1 inhibitors have made breakthroughs in the treatment of lung cancer [28]. From the first-line and second-line therapy to consolidation therapy, immunotherapy has shown great potential in the individualized and precise treatment of lung cancer [29]. Malignant tumor cells can express PD-L1 through two mechanisms: one is congenital immune resistance, that is, in some tumors, component carcinogenic signal transduction directly upregulates the expression of PD-L1 on all tumor cells, which is a genetic event and has nothing to do with inflammatory stimulation [30–32]. The second is adaptive immune resistance, that is, the expression of PD-L1 induced by inflammatory signals (such as interferon *γ*) generated by antitumor immune response [33]. Pembrolizumab is a humanized IgG4 monoclonal antibody against PD-1. This is the first phase B clinical study to evaluate the efficacy and safety of pembrolizumab in advanced NSCLC. It was found that the effect was better in patients with elevated PD-L1 expression [34].

RETRACTED

A total of 14 RCTS of pembrolizumab treatment for NSCLC were included in this study. Following the principles of Cochrane systematic evaluation, meta-analysis was used to analyze indicators such as OS, PFS, 1-year survival rate, and incidence of common adverse reactions [35]. Meta-analysis results showed that pembrolizumab combined with chemotherapy improved 1-year survival rate and prolonged OS, with statistically significant differences compared with chemotherapy alone, while complete response rate, PFS, and chemotherapy alone showed no statistically significant differences. Relevant studies [36–38] also showed that pembrolizumab combined with chemotherapy had a higher proportion of grade 3 and 4 leukopenia, rash, and infusion reaction than chemotherapy alone, and the difference was statistically significant, but there was no increase in the mortality rate. Therefore, pembrolizumab is effective and safe.

The following are some of the restrictions that apply to this study: (1) The criteria for what constitutes a positive PD-L1 test, known as the cutoff value, may vary [39]. The weakness of this work is that it does not conduct a subgroup analysis of shortened values, which may contribute to an increase in research bias. (2) Responses to immunotherapy might vary depending on the molecular profile of non-small-cell lung cancer [40].

RETRACTED

In conclusion, the administration of pembrolizumab in conjunction with chemotherapy for patients with NSCLC may enhance treatment effectiveness. This occurs even if the frequency of certain adverse responses has risen; nevertheless, it does not raise the mortality rate. Therefore, pembrolizumab may be tolerated and should be used in clinical settings on a more extensive scale.

## Figures and Tables

**Figure 1:** Flow chart of the literature screening.

**Figure 2:** Literature quality evaluation chart. (a) Risk of bias graph; (b) risk of bias summary.

**Figure 3:** (a–d) Funnel plot of literature publication bias.

**Figure 4:** Meta-analysis of one-year survival rate between two groups.

**Figure 5:** Meta-analysis of overall response rate between two groups.

**Figure 6:** Meta-analysis of progression-free survival between two groups.

**Figure 7:** Meta-analysis of overall survival between two groups.

**Figure 8:** Meta-analysis of incidence of coincidences between two groups.

**Table 1:** Basic clinical features of 14 literatures were included in our study.

Study	Age	Gender (man)	Hospitalization days	Experimental group (*N*)	Control group (*N*)	NOS score	Research type
Reck M [11]	63.25 ± 12.2	42.25%	6.8 ± 1.1	200/305	105/305	7	RCT
Garon EB [12]	65.55 ± 13.4	68.12%	6.2 ± 1.3	315/495	278/495	7	RCT
Reck M [13]	63.32 ± 14.5	46.72%	5.4 ± 3.9	167/305	158/305	8	RCT
Goldberg SB [14]	67.15 ± 13.5	45.12%	6.9 ± 4.9	33/52	28/52	7	RCT
Eichhorn F [15]	62.85 ± 8.5	51.89%	9.8 ± 3.4	21/30	15/30	8	RCT
Amrane K [16]	64.26 ± 10.2	63.45%	5.2 ± 5.1	67/108	54/108	7	RCT
Jabbour SK [17]	62.62 ± 12.1	68.10%	6.9 ± 2.1	12/21	9/21	7	RCT
Middleton G [18]	62.61 ± 13.5	49.75%	5.9 ± 1.4	78/112	56/112	7	RCT
Herbst RS [19]	57.15 ± 14.5	59.23%	6.4 ± 4.1	51/92	41/92	7	RCT
Lisberg A [20]	66.22 ± 15.1	57.22%	7.8 ± 1.5	14/25	11/25	8	RCT
Eichhorn F [21]	61.35 ± 8.1	54.16%	6.1 ± 5.9	10/15	5/15	7	RCT
Hellmann MD [22]	67.15 ± 16.0	67.34%	7.5 ± 1.6	322/601	255/601	7	RCT
Weiss GJ [23]	58.11 ± 8.6	49.34%	5.0 ± 5.6	39/49	28/49	9	RCT
Hui R [24]	66.34 ± 6.4	54.12%	6.4 ± 1.7	68/101	56/101	8	RCT

## References

[1] De Ruysscher D., Faivre-Finn C., Nackaerts K. (2020). Recommendation for supportive care in patients receiving concurrent chemotherapy and radiotherapy for lung cancer. *Annals of Oncology*.

[2] Dafni U., Tsourti Z., Vervita K., Peters S. (2019). Immune checkpoint inhibitors, alone or in combination with chemotherapy, as first-line treatment for advanced non-small cell lung cancer. A systematic review and network meta-analysis. *Lung Cancer*.

RETRACTED

[3] El-Hussein A., Manoto S. L., Ombinda-Lemboumba S., Alrowaili Z. A., Mthunzi-Kufa P. (2021). A review of chemotherapy and photodynamic therapy for lung cancer treatment. *Anti-Cancer Agents in Medicinal Chemistry*.

[4] Griesinger F., Korol E. E., Kayaniyil S., Varol N., Ebner T., Goring S. M. (2019). Efficacy and safety of first-line carboplatin-versus cisplatin-based chemotherapy for non-small cell lung cancer: a meta-analysis. *Lung Cancer*.

[5] Wang C., Qiao W., Jiang Y. (2020). The landscape of immune checkpoint inhibitor plus chemotherapy versus immunotherapy for advanced non-small-cell lung cancer: a systematic review and meta-analysis. *Journal of Cellular Physiology*.

[6] Curtis L. T., Frieboes H. B. Modeling of combination chemotherapy and immunotherapy for lung cancer.

[7] Wen L., Tong F., Zhang R., Chen L., Huang Y., Dong X. (2021). The research progress of PD-1/PD-L1 inhibitors enhancing radiotherapy efficacy. *Frontiers in Oncology*.

[8] Jimbu L., Mesaros O., Popescu C. (2021). Is there a place for PD-1-PD-L blockade in acute myeloid leukemia?. *Pharmaceuticals (Basel)*.

[9] Nie M., Liu Y., Li X. X. (2019). PD-1/PD-L pathway potentially involved in ITP immunopathogenesis. *Thrombosis and Haemostasis*.

[10] Grecea M., Soritau O., Dulf D., Ciuleanu T. E., Zdrenghea M. (2021). Potential biomarkers for the efficacy of PD-1-PD-L blockade in cancer. *Oncotargets and Therapy*.

[11] Reck M., Rodríguez-Abreu D., Robinson A. G. (2016). Pembrolizumab versus chemotherapy for PD-L1-positive non-small-cell lung cancer. *The New England Journal of Medicine*.

[12] Garon E. B., Rizvi N. A., Hui R. (2015). Pembrolizumab for the treatment of non-small-cell lung cancer. *The New England Journal of Medicine*.

[13] Reck M., Rodríguez-Abreu D., Robinson A. G. (2021). Five-year outcomes with pembrolizumab versus chemotherapy for metastatic non-small-cell lung cancer with PD-L1 tumor proportion score ≥ 50%. *Journal of Clinical Oncology*.

[14] Goldberg S. B., Gettinger S. N., Mahajan A. (2016). Pembrolizumab for patients with melanoma or non-small-cell lung cancer and untreated brain metastases: early analysis of a non-randomised, open-label, phase 2 trial. *The Lancet Oncology*.

[15] Eichhorn F., Klotz L. V., Bischoff H. (2019). Neoadjuvant anti-programmed death-1 immunotherapy by pembrolizumab in resectable nodal positive stage II/IIIa non-small-cell lung cancer (NSCLC): the NEOMUN trial. *BMC Cancer*.

[16] Amrane K., Geier M., Corre R. (2020). First-line pembrolizumab for non–small cell lung cancer patients with PD-L1 ≥50% in a multicenter real-life cohort: The PEMBREIZH study. *Cancer Medicine*.

RETRACTED

[17] Jabbour S. K., Berman A. T., Decker R. H. (2020). Phase 1 trial of pembrolizumab administered concurrently with chemoradiotherapy for locally advanced non-small cell lung cancer: a nonrandomized controlled trial. *JAMA Oncology*.

[18] Middleton G., Brock K., Savage J. (2020). Pembrolizumab in patients with non-small-cell lung cancer of performance status 2 (PePS2): a single arm, phase 2 trial. *The Lancet Respiratory Medicine*.

[19] Herbst R. S., Arkenau H. T., Santana-Davila R. (2019). Ramucirumab plus pembrolizumab in patients with previously treated advanced non-small-cell lung cancer, gastro-oesophageal cancer, or urothelial carcinomas (JVDF): a multicohort, non-randomised, open-label, phase 1a/b trial. *The Lancet Oncology*.

[20] Lisberg A., Cummings A., Goldman J. W. (2018). A phase II study of pembrolizumab in EGFR-mutant, PD-L1+, tyrosine kinase inhibitor naive patients with advanced NSCLC. *Journal of Thoracic Oncology*.

[21] Eichhorn F., Klotz L. V., Kriegsmann M. (2021). Neoadjuvant anti-programmed death-1 immunotherapy by pembrolizumab in resectable non-small cell lung cancer: first clinical experience. *Lung Cancer*.

[22] Hellmann M. D., Jänne P. A., Opyrchal M. (2021). Entinostat plus pembrolizumab in patients with metastatic NSCLC previously treated with anti-PD-(L)1 therapy. *Clinical Cancer Research*.

[23] Weiss G. J., Waypa J., Blaydorn L. (2017). A phase Ib study of pembrolizumab plus chemotherapy in patients with advanced cancer (PembroPlus). *British Journal of Cancer*.

[24] Hui R., Garon E. B., Goldman J. W. (2017). Pembrolizumab as first-line therapy for patients with PD-L1-positive advanced non-small cell lung cancer: a phase 1 trial. *Annals of Oncology*.

[25] Yang S. J., Huang C. H., Wang C. H., Shieh M. J., Chen K. C. (2020). The synergistic effect of hyperthermia and chemotherapy in magnetite nanomedicine-based lung cancer treatment. *International Journal of Nanomedicine*.

[26] Huang M., Lopes G. L., Insinga R. P. (2019). Cost-effectiveness of pembrolizumab versus chemotherapy as first-line treatment in PD-L1-positive advanced non-small-cell lung cancer in the USA. *Immunotherapy*.

[27] Jin Y., Wang Y., Liu X. (2020). Synergistic combination chemotherapy of lung cancer: cisplatin and doxorubicin conjugated prodrug loaded, glutathione and pH sensitive nanocarriers. *Drug Design, Development and Therapy*.

[28] Wang B., Hu W., Yan H. (2021). Lung cancer chemotherapy using nanoparticles: enhanced target ability of redox-responsive and pH-sensitive cisplatin prodrug and paclitaxel. *Biomedicine & Pharmacotherapy*.

[29] Shiraishi T., Oda K., Yamasaki K. (2022). Risk factors for in-hospital mortality in patients with advanced lung cancer with interstitial pneumonia undergoing systemic chemotherapy: a retrospective and observational study using a nationwide administrative database in Japan. *Thorac Cancer*.

RETRACTED

[30] Chang Q., Xu J., Qiang H. (2021). _EGFR_ tyrosine kinase inhibitor (TKI) combined with concurrent or sequential chemotherapy for patients with advanced lung cancer and gradual progression after first-line _EGFR_ -TKI therapy: a randomized controlled study. *Clinical Lung Cancer*.

[31] Zhang M., Liu D., Zhou H. (2021). Intestinal flora characteristics of advanced non-small cell lung cancer in China and their role in chemotherapy based on metagenomics: a prospective exploratory cohort study. *Thorac Cancer*.

[32] Horiuchi K., Sato T., Kuno T. (2021). Platinum-doublet chemotherapy as second-line treatment for relapsed patients with small-cell lung cancer: a systematic review and meta-analysis. *Lung Cancer*.

[33] Zhang H., Yang J., Deng Y. M. (2019). Multiple-line chemotherapy and tyrosine kinase inhibitor treatment in patients with advanced lung cancer. *Combinatorial Chemistry & High Throughput Screening*.

[34] Tong Y., Wen J., Yang T. (2021). Clinical efficacy and safety of tanreqing injection combined with antibiotics versus antibiotics alone in the treatment of pulmonary infection patients after chemotherapy with lung cancer: a systematic review and meta-analysis. *Phytotherapy Research*.

[35] Qin W., Hu L., Zhang X. (2019). The diverse function of PD-1/PD-L pathway beyond cancer. *Frontiers in Immunology*.

[36] Zhang P. P., Wang J., Ding D. Z., Zhang L., Cheng C., Chen D. K. (2021). Efficacy and safety of PD-1/PD-L1 inhibitors combined with CTLA-4 inhibitor versus chemotherapy for advanced lung cancer: a meta-analysis. *Medicine (Baltimore)*.

[37] Li M., Chen R., Ji B. (2021). Role of ERCC5 polymorphisms in non-small cell lung cancer risk and responsiveness/toxicity to cisplatin-based chemotherapy in the Chinese population. *Oncology Reports*.

[38] Gong W. J., Ma L. Y., Hu L. (2019). STAT3 rs 4796793 contributes to lung cancer risk and clinical outcomes of platinum-based chemotherapy. *International Journal of Clinical Oncology*.

[39] Ito R., Tsukioka T., Izumi N. (2022). Lymph node metastasis location and postoperative adjuvant chemotherapy in patients with pN1 stage IIB non-small cell lung cancer. *In Vivo*.

[40] Nakashima K., Hata K., Hotta T. (2021). Ability of the Glasgow Prognostic Score to predict the tolerability and efficacy of platinum-combination chemotherapy among elderly patients with advanced non-small cell lung cancer. *The Journal of Medical Investigation*.

